The article "Efficacy and safety of atypical antipsychotic drug treatment for dementia: a systematic review and meta-analysis" was retracted in 2016. Reasons: errors in the data; errors in the methods.

# Efficacy and safety of atypical antipsychotic drug treatment for dementia: a systematic review and meta-analysis

**DOI:** 10.1186/s13195-015-0102-9

**Published:** 2015-04-20

**Authors:** Lin Tan, Lan Tan, Hui-Fu Wang, Jun Wang, Chen-Chen Tan, Meng-Shan Tan, Xiang-Fei Meng, Chong Wang, Jin-Tai Yu

**Affiliations:** College of Medicine and Pharmaceutics, Ocean University of China, Qingdao, 266000 China; Department of Neurology, Qingdao Municipal Hospital, School of Medicine, Qingdao University, Qingdao, 266071 China; Department of Neurology, Qingdao Municipal Hospital, Nanjing Medical University, Nanjing, 210000 China

## Abstract

**Introduction:**

A wide variety of atypical antipsychotic drugs (risperidone, olanzapine, quetiapine, aripiprazole, ziprasidone and clozapine) are widely used in the management of neuropsychiatric symptoms, which are commonly seen in dementia, but results from randomised controlled trials (RCTs) on the efficacy and safety of these agents are conflicting. We aimed to quantify the efficacy and safety of atypical antipsychotic drugs on neuropsychiatric symptoms in dementia patients.

**Methods:**

PubMed, EMBASE, the Cochrane Controlled Trials Register and the Cochrane Database of Systematic Reviews for reports published before August 2014 were searched for eligible randomized controlled trials of atypical antipsychotic drugs therapy in patients with psychotic symptoms of dementia. Two reviewers independently assessed the quality of the trials and extracted information.

**Results:**

Overall, 23 relevant RCTs with 5,819 participants were identified. This meta-analysis demonstrated a significant efficacy of atypical antipsychotics on psychiatric symptoms and cognitive functions compared to placebo. In the meta-analysis, the weighted mean differences (WMDs) in change scores for psychiatric symptoms were in favor of aripiprazole (−4.4, 95% confidence interval (CI) – 7.04 to −1.77) and risperidone (−1.48, 95% CI −2.35 to −0.61) compared to placebo. In cognitive effects, WMDs in change scores for the Clinical Global Impression-Change (CGI-C) were in favor of aripiprazole, risperidone, olanzapine and quetiapine which ranged from a −0.30 points mean difference (95% CI:-0.59 to −0.01) in the aripiprazole trials to −0.43 (95% CI:-0.62 to −0.25) in the risperidone group. Patients receiving atypical antipsychotics showed no difference in risk for injuries or falls (*P* > 0.05), significantly higher risks (*P* < 0.05) for somnolence, urinary tract infection, edema and abnormal gait. However, there was no significant evidence for death reported.

**Conclusion:**

Aripiprazole and risperidone are able to improve psychiatric symptoms and slow decline in cognition function at average 12 weeks in patients with neuropsychiatric symptoms of dementia. However, high adverse events may offset the efficacy of atypical antipsychotics in dementia.

The article "Efficacy and safety of atypical antipsychotic drug treatment for dementia: a systematic review and meta-analysis" was retracted in 2016. Reasons: errors in the data; errors in the methods.

**Electronic supplementary material:**

The online version of this article (doi:10.1186/s13195-015-0102-9) contains supplementary material, which is available to authorized users.

## Introduction

The global prevalence of dementia is as high as 24 million cases worldwide and has been predicted to quadruple by the year 2050. Dementia causes unestimated healthcare costs per year [1]. Neuropsychiatric symptoms rather than cognitive dysfunction or functional impairment have been suggested to impose the greatest burden on family caregivers, and to predict caregivers’ decisions to institutionalize patients with dementia. Interventions targeting improving neuropsychiatric symptoms could therefore have a tremendous impact on patients, caregivers and society. There are multiple classes of pharmacological agents in use for neuropsychiatric symptoms, especially antipsychotics. The typical antipsychotic medications (for example, haloperidol or thioridazine), with or without psychosocial and environmental interventions, are frequently used to treat symptoms that occur in a majority of older patients with dementia during their illness courses, and have been the mainstay of psychopharmacologic treatment during the last several decades [2]. Interestingly, the atypical antipsychotics (that is, risperidone, olanzapine, quetiapine, aripiprazole, ziprasidone and clozapine) generally have replaced conventional antipsychotics [3]. Atypical antipsychotics are approved for marketing and labeling by the US Food and Drug Administration for treating schizophrenia, bipolar disorder and depression under drug-specific circumstances [4]. To date, the use of atypical antipsychotic medications is rapidly increasing in the USA. They have been considered the preferred pharmacologic treatment for behavioral disturbances associated with dementia because evidence from clinical trials perceived safety advantages compared with other medications and expert clinical opinion [5].

The role of currently available atypical antipsychotics for dementia has been controversial, however, with some national formularies restricting their use and health economists questioning whether the small clinical effects are economically worthwhile. Moreover, the efficacy of ziprasidone and clozapine in the treatment of dementia has also been heavily debated. In addition, high dropout rates and numerous adverse events have been observed in randomized clinical trials of these agents. Besides, safety concerns have been raised about the atypical antipsychotics. Some clinical trials and meta-analyses have evaluated the efficacy and safety of these drugs on neuropsychiatric symptoms, but have had conflicting findings [6]. We thus performed a systematic review and meta-analysis to clarify the efficacy and safety of these atypical antipsychotics for neuropsychiatric symptoms in dementia patients. We sought to elaborate on previous reviews articles by including a broad spectrum of outcome measures, and to determine whether these drugs have different degrees of efficacy on psychiatric symptoms and cognitive functions of dementia. Previous systematic reviews or meta-analyses have been incomplete in this regard.

The article "Efficacy and safety of atypical antipsychotic drug treatment for dementia: a systematic review and meta-analysis" was retracted in 2016. Reasons: errors in the data; errors in the methods.

## Methods

### Search strategy

The search strategy was described in detail. Briefly, we systematically searched PubMed, EMBASE, the Cochrane Controlled Trials Register and the Cochrane Database of Systematic Reviews for reports published before August 2014. The search criteria combined three separate domains: condition (dementia), intervention (risperidone, olanzapine, quetiapine, aripiprazole, ziprasidone, clozapine) and symptoms (behavioral and psychological symptoms of dementia, BPSD, neuropsychiatric symptoms, behavior). We included studies reporting overall symptoms of agitation, psychosis or aggression. Terms were searched in titles and abstracts. We retrieved English-language articles for review, and also collected additional references from bibliographies of reviews, original research articles and other articles of interest. Pharmaceutical manufacturers were queried and information was requested as needed.

Two investigators independently reviewed all pertinent articles using predetermined inclusion criteria. Trials were selected for inclusion if they met all of the following criteria: parallel group, double-blind, placebo-controlled, randomized controlled trials (RCTs); patients had psychiatric symptoms with Alzheimer’s disease (AD), vascular dementia, mixed dementia or a primary dementia according to the *Diagnostic and Statistical Manual of Mental Disorders – Fourth Edition* [7]; and the number of patients randomized and at least one outcome measure or adverse event were obtainable.

### Trials selection

We selected double-blind, placebo-controlled RCTs comparing atypical antipsychotics with placebo that used the scales. Generally, trials of specific drugs used different outcomes from trials of other drugs. The Brief Psychiatric Rating Scale (BPRS) [8] and the Neuropsychiatric Inventory (NPI) [9] are used mainly for aripiprazole trials, olanzapine trials, some quetiapine trials and few risperidone trials. The Behavioral Pathology in Alzheimer’s Disease Rating Scale (BEHAVE-AD) [10] and the Cohen-Mansfield Agitation Inventory (CMAI) [11] were generally used for risperidone trials. The Clinical Global Impression – Change (CGI-C) and the Clinical Global Impression – Severity (CGI-S) [12] were also used as clinical outcomes in some trials. We used the NPI-total score, BPRS-total score and BEHAVE-AD score as the psychiatric symptoms, while the CGI-C and Minimum Mental State Examination (MMSE) were used as the cognitive functions. There is little clinical trial evidence for the efficacy of ziprasidone and clozapine [6].

The article "Efficacy and safety of atypical antipsychotic drug treatment for dementia: a systematic review and meta-analysis" was retracted in 2016. Reasons: errors in the data; errors in the methods.

### Data retrieval

Information extracted included design characteristics, selection criteria (dementia diagnoses and presence of psychosis of dementia), medication doses, trial durations (6 to 26 weeks), age, race, gender, baseline cognitive scores, baseline neuropsychiatric symptoms and numbers randomized. The minimum baseline score for the NPI-total and the BPRS-total was 20 while that for the BEHAVE-AD was 15. For each trial, two reviewers were blinded to the authors and journal, and independently abstracted data. The mean change of scale scores and standard deviations for the mean change were extracted. For standard deviations that were not reported directly, we sought them from the authors or calculated them from standard errors, confidence intervals (CIs) or *P* values that relate to the difference between means in two groups according to the *Cochrane Handbook for Systematic Reviews of Interventions* [13]. Studies were excluded if the mean change of scale total scores were not available. Moreover, if there were duplicate publications from the same population, only one of the trials that reported the mean change of scale total score and standard deviation was included; others were excluded. Outcomes and adverse events data were from the intent-to-treat or last-observation-carried-forward samples. Discrepancies in the collected data were discussed, and if consensus was not reached a third reviewer was the final arbitrator.

### Statistical analysis

Meta-analyses were performed using Review Manager V.5.2 software (Review Manager, Version 5.2, Copenhagen: The Nordic Cochrane Centre, The Cochrane Collaboration, Denmark). Combining the scales in an overall summary estimate, we calculated weighted mean differences (WMDs) and 95% CIs for changes from baseline for continuous data. For dichotomous dropouts and adverse events, we conducted an analysis of the odds ratio (OR), absolute risk differences with 95% CI and *P* values to assess the safety of the study drug. A random-effects model was applied to assess the effect sizes for each treatment–placebo comparison in our study.

Because there were few dose-ranging trials and sparse outcomes for adverse events, and to avoid multiple comparisons with the same placebo group, we combined dosage groups within each trial to make one contrast with placebo according to the *Cochrane Handbook for Systematic Reviews of Interventions*. The degree of heterogeneity was assessed by visual inspection, and by a chi-square test combined with the *I*^2^ method. The *I*^2^ statistic approximates the proportion of total variation in the effect size estimates that is the result of heterogeneity rather than sampling error. Values of α error *P* <0.20 and *I*^2^ > 50% were regarded as indicators of heterogeneity of outcomes.

The article "Efficacy and safety of atypical antipsychotic drug treatment for dementia: a systematic review and meta-analysis" was retracted in 2016. Reasons: errors in the data; errors in the methods.

## Results

### Characteristics of included trials

The results of the search process are depicted in the flowchart (Figure 1). Of 886 articles identified, three aripiprazole articles [14-16], five olanzapine articles [17-21], seven quetiapine articles [17,19,22-26] and eight risperidone articles [17,19,20,27-31] met all review criteria. All studies were RCTs and were performed mainly in North American and European countries. Baseline characteristics were similar between intervention and placebo groups in all of the trials. The included studies were all randomized parallel trials for which the duration was 6 to 26 weeks. In all, 13 trials compared one fixed dose of medicine and placebo, and five trials were dose ranging. Among these dose-ranging studies, three used more than one dose compared with a single placebo group. These trials included 3,927 patients in the medicine treatment group and 1,892 participants in the placebo treatment group. The mean ages of patients in the medicine treatment groups ranged from 77.3 to 84.2 years. The mean baseline MMSE scores ranged from 4.8 to 15.7. Additional file 1 presents characteristics of these studies and populations in more detail.

**Figure 1:** **Flowchart of randomized controlled trials included and excluded in the meta-analysis.** RCT, randomized controlled trial.

### Bias risk assessment

Although all included trials were randomized, double blinded and placebo controlled, specification of randomization and allocation concealment methods were different from each other. The randomization was conducted according to a computerized randomization schedule among nine trials, four reports specified the varied methods of randomization and the other 14 reports did not give detailed information although they involved noted randomization. Besides, efficacy outcomes of all trials were analyzed by intent-to-treat data with the last-observation-carried-forward method for minimizing effects of attrition bias. A funnel plot did not show evidence of selection bias with symmetry around the mean overall effect.

The article "Efficacy and safety of atypical antipsychotic drug treatment for dementia: a systematic review and meta-analysis" was retracted in 2016. Reasons: errors in the data; errors in the methods.

### Psychiatric symptoms

For psychiatric symptoms, 15 studies measured and reported the mean change in NPI-total score from baseline to end point for intervention compared with placebo: three studies on aripiprazole [14-16], five studies on olanzapine [17-21], two studies on quetiapine (50 mg) [17,19], three studies on quetiapine (100 mg) [22,23,25] and two studies on risperidone [17,19]. All of these studies included participants with moderate to severe dementia. NPI-total scores were only significant for aripiprazole by meta-analysis in the available data (−4.4, 95% CI = −7.04 to −1.77). In the quetiapine trials, the differences by meta-analysis were −4.3 (95% CI = −8.81 to 0.21) for the 50 mg daily group and −0.12 (95% CI = −1.74 to 1.50) for the 100 mg daily group. In addition, the difference between the olanzapine group and placebo was −2.61 (95% CI = −5.23 to −0.00) (Figure 2). The pooled study NPI-total score was −1.68, which was of great significance (*P* = 0.004). Fourteen trials used the BPRS-total score: three studies on aripiprazole [14-16], five studies on olanzapine [17-21], two studies on quetiapine (50 mg) [17,19], two studies on quetiapine (100 mg) [23,25] and two studies on risperidone [17,19]. The score was only significant for aripiprazole by meta-analysis in the available data (95% CI = −3.44 to −0.62). In the quetiapine trials, the differences by meta-analysis were −1.82 (95% CI = −4.00 to 0.36) for the 50 mg daily group and −2.23 (95% CI = −4.83 to 0.38) for the 100 mg daily group. In addition, the difference between the olanzapine group and placebo was −0.60 (95% CI = −1.98 to 0.78) (Figure 3). Only four risperidone trials reported changes in the BEHAVE-AD score [27-30]. The BEHAVE-AD scores were significant for risperidone by meta-analysis in the available data. The WMDs by meta-analysis were −1.48 (95% CI = −2.35 to −0.61) (Figure 4). Furthermore, the effects with four drugs (risperidone, olanzapine, quetiapine, aripiprazole) on specific psychosis subscales of the BPRS (see Additional file 2), NPI (see Additional file 3) or BEHAVE-AD (see Additional file 4) were analyzed. There were no significant effects by meta-analysis for three aripiprazole trials, three olanzapine trials, one risperidone trial and one quetiapine trial on the NPI psychosis subscales (WMD = −0.42, 95% CI = −0.91 to 0.08, *P* = 0.29). However, aripiprazole trials alone showed a significant effect on NPI psychosis subscales (WMD = −0.88, 95% CI = −1.61 to −0.16, *P* = 0.02). For aripiprazole, the BPRS psychosis subscale scores by meta-analysis were not significant (WMD = −0.23, 95% CI = −0.60 to 0.08, *P* = 0.23). There was a significant effect by meta-analysis with risperidone on the BEHAVE-AD psychosis subscale from four trials (WMD = −0.84, 95% CI = −1.24 to −0.44, *P* <0.0001). The quality of reports for all included studies was appraised with GRADE software (Grading of Recommendations Assessment, Development and Evaluation, Version 3.6, Hamilton, Canada), and the outcome is presented in Additional files 5, 6 and 7.

The article "Efficacy and safety of atypical antipsychotic drug treatment for dementia: a systematic review and meta-analysis" was retracted in 2016. Reasons: errors in the data; errors in the methods.

**Figure 2:** **Forest plot for efficacy of the Neuropsychiatric Inventory-total score on dementia patients in subgroup analyses.** Data type, continuous; effect measure, weighted mean difference; analysis model, fixed effects; statistical method, inverse variance. CI, confidence interval; SD, standard deviation.

**Figure 3:** **Forest plot for efficacy of the Brief Psychiatric Rating Scale-total score on dementia patients in subgroup analyses.** Data type, continuous; effect measure, weighted mean difference; analysis model, fixed effects; statistical method, inverse variance. CI, confidence interval; SD, standard deviation.

**Figure 4:** **Forest plot for efficacy of the Behavioral Pathology in Alzheimer’s Disease Rating Scale score on dementia patients in subgroup analyses.** Data type, continuous; effect measure, weighted mean difference; analysis model, fixed effects; statistical method, inverse variance. CI, confidence interval; SD, standard deviation.

### Cognitive functions

Thirteen studies measured and reported the mean change in CGI-C from baseline to end point for intervention compared with placebo: one study on aripiprazole [15], three studies on olanzapine [17,19,21], five studies on quetiapine [19,22-25] and four studies on risperidone [17,19,27-30]. CGI-C scores were all significant for these trials by meta-analysis in the available data. The difference between the pooled group and placebo was −0.36 (95% CI = −0.47 to −0.25) (Figure 5). Furthermore, 13 trials reported MMSE change scores: three aripiprazole contrasts [14-16], three olanzapine contrasts [17,18,20], two risperidone contrasts [17,20] and five quetiapine contrasts [19,22-25]. The overall effect of drugs compared with placebo was a WMD of −0.34 (95% CI = −0.65 to −0.03, *P* = 0.03) in favor of placebo. The three aripiprazole trials showed statistical significance of MMSE in favor of placebo (WMD = −0.99, 95% CI = −1.65 to −0.33, *P* = 0.003) (Figure 6). The quality of reports for all included studies was appraised with GRADE software. The outcome is presented in Additional files 8 and 9.

**Figure 5:** **Forest plot for Clinical Global Impression – Change subscale scores on dementia patients in subgroup analyses.** Data type, continuous; effect measure, weighted mean difference; analysis model, fixed effects; statistical method, inverse variance. CI, confidence interval; SD, standard deviation.

The article "Efficacy and safety of atypical antipsychotic drug treatment for dementia: a systematic review and meta-analysis" was retracted in 2016. Reasons: errors in the data; errors in the methods.

**Figure 6:** **Forest plot for Minimum Mental State Examination in dementia patients.** Data type, continuous; effect measure, weighted mean difference; analysis model, fixed effects; statistical method, inverse variance. CI, confidence interval; SD, standard deviation.

### General assessment of atypical antipsychotic drugs

#### Aripiprazole

The three aripiprazole trials retrieved were designed similarly, with similar selection criteria – AD with psychosis and 10-week treatment durations – and the same primary and secondary outcomes – that is, BPRS, NPI, CGI-S and CMAI. Two were nursing home trials and one was an outpatient trial. One trial was a dose-ranging trial including 2, 5 and 10 mg/day [15]. Significant effects by meta-analysis were observed on the BPRS-total and NPI-total change scores (WMD = −4.4, 95% CI = −7.04 to −1.77, *P* = 0.001; WMD = −2.03, 95% CI = −3.44 to −0.62, *P* = 0.005). A significant effect by meta-analysis on the CMAI was observed but was based on only the two nursing home trials (WMD = −4.73, 95% CI = −7.43 to −2.03, *P* = 0.0006). Global clinical ratings were reported only as continuous outcomes with a one-point to seven-point range and not as categorical or individual response-based outcomes. The CGI-S was significant in favor of aripiprazole by meta-analysis (WMD = −0.16, 95% CI = −3.0 to −0.03, *P* = 0.02). The heterogeneity among the study was mild (*I*^2^ = 0%).

#### Olanzapine

Among the five olanzapine trials, four trials retrieved were designed with similar selection criteria – AD with psychosis, 6-week to 12-week treatment durations – and the same primary outcomes – that is, BPRS and NPI. Two were nursing home trials and three were outpatient trials. Three trials chose patients with psychotic and behavioral symptoms. Other two trials focused on patients with psychosis, aggression or agitation. Two trials were dose-ranging trials including 5, 10 and 15 mg/day and 5 and 7.5 mg/day respectively. We only chose the average 5 mg/day group for meta-analysis.

Among these five trials, there were nonsignificant effects by meta-analysis on the BPRS and NPI (WMD = −0.6, 95% CI = −1.98 to 0.78, *P* = 0.40; WMD = −2.61, 95% CI = −5.23 to 0.00, *P* = 0.05;respectively).

#### Quetiapine

The designs, selection criteria and outcomes scales differed substantially among the seven quetiapine trials and we combined the same dose group for efficacy outcomes. One study enrolled primarily nursing home patients with psychosis in patients with probable/possible AD and assessed other psychopathology and social and daily functioning [23]. Four trials chose patients with a primary dementia, AD, vascular dementia or mixed dementia, mainly manifesting agitation severe enough to require an antipsychotic. Among the four trials, a smaller trial chose nursing home patients with AD and agitation and compared quetiapine treatment with rivastigmine and placebo [26]. The other two trials focused on the behavioral and psychological symptoms of dementia patients [17,24].

The article "Efficacy and safety of atypical antipsychotic drug treatment for dementia: a systematic review and meta-analysis" was retracted in 2016. Reasons: errors in the data; errors in the methods.

Two trials showed no significant effect for the 50 mg/day quetiapine treatment groups on the BPRS and NPI (WMD = −1.82, 95% CI = −4.00 to 0.36, *P* = 0.10; WMD = −4.3, 95% CI = −8.81 to 0.21, *P* = 0.06; respectively). Three trials showed no statistically significant effect for the 100 mg/day quetiapine treatment groups on the BPRS and NPI (WMD = −0.12, 95% CI = −1.74 to 1.50, *P* = 0.89; WMD = −2.23, 95% CI = −4.83 to 0.38, *P* = 0.09; respectively).

#### Risperidone

Among the eight risperidone trials, four were similarly designed in that they selected nursing home patients with dementia and aggression, had a minimum score on the BEHAVE-AD of ≥8 and were treated for an average 12 weeks. Three trials enrolled AD patients with psychotic and behavioral symptoms. Schneider and colleagues’ trial selected patients with psychosis. These eight trials used similar primary efficacy outcomes; that is, the BEHAVE-AD and CMAI. The CGI-C, CGI-S, NPI and BPRS were also used as secondary outcomes in some trials.

Among the four trials using the BEHAVE-AD, there was overall significant improvement with risperidone (WMD = −1.48, 95% CI = −2.35 to −0.61, *P* = 0.0008) and on the CMAI used in three trials (WMD = −3.00, 95% CI = −4.22 to −1.78, *P* <0.00001). There was a statistically significant effect overall by meta-analysis on the CGI-S in two trials as a continuous variable (WMD = −0.39, 95% CI = −0.58 to −0.20, *P* <0.0001). However, no significant difference was observed for the NPI or BPRS score.

### Safety

#### Adverse events

Adverse events were inconsistently reported among the trials; most did not report adverse events occurring less than 20% of the time, and potentially significant adverse events could not be counted from all trials. Somnolence, falls, injury, edema and urinary tract infections were mostly reported from the trials. Adverse events are summarized by the numbers of trials for which the event was reported and the odds ratio for the event (Table 1). The quality of reports of all included studies was appraised with GRADE software, and the outcome is presented in Additional file 10.

**Table 1:** **Odds ratios by meta-analysis of adverse effects in atypical antipsychotics compared with placebo**

		**Somnolence**	**Injuries or falls**	**Abnormal gait**	**Edema**	**Urinary infection**	**Stroke**
Aripiprazole	OR	3.51	0.86	5.04	0.93	1.20	1.58
	(95% CI)	(1.64, 7.5)	(0.58, 1.28)	(0.58, 43.81)	(0.38, 2.27)	(0.78, 1.87)	(0.38, 6.55)
Olanzapine	OR	3.61	1.13	3.84	0.52	6.93	3.93
	(95% CI)	(1.83, 7.13)	(0.72, 1.76)	(1.64, 8.95)	(0.16, 1.69)	(1.33, 35.96)	(0.62, 25.10)
Risperidone	OR	3.57	0.85	1.21	0.49	2.28	4.53
	(95% CI)	(2.72, 4.67)	(0.68, 1.08)	(0.73, 1.99)	(0.30, 0.78)	(1.58,3.30)	(1.75, 11.72)
Quetiapine	OR	5.88	0.86	1.98	1.51	1.90	1.13
	(95% CI)	(2.39, 14.47)	(0.57, 1.29)	(0.73, 5.39)	(0.55, 4.19)	(0.95, 3.8)	(0.36, 3.56)

CI, confidence interval; OR, odds ratio.

The article "Efficacy and safety of atypical antipsychotic drug treatment for dementia: a systematic review and meta-analysis" was retracted in 2016. Reasons: errors in the data; errors in the methods.

#### Somnolence

The 13 available comparisons all showed increased risk for somnolence, and all of them were statistically significant. The odds ratio by meta-analysis was 3.7 (95% CI = 2.94 to 4.66, *P* <0.00001) with significant heterogeneity. Significant risk differences were found among aripiprazole (OR = 3.51, 95% CI = 1.64 to 7.50), olanzapine (OR = 3.61, 95% CI = 1.83 to 7.13) and quetiapine (OR = 5.88, 95% CI = 2.39 to 14.47) with small heterogeneity (*I*^2^ = 0%).

#### Injury or falls

Outcomes are consistent in the 15 contrasts that provided data for injury/accidental injury and falls. They did not show an increase or decrease in risk overall or in the result of a particular drug or trial (OR = 0.89, 95% CI = 0.75 to 1.05, *P* = 0.17).

#### Abnormal gait

There was an overall increased risk for abnormal gait in the pooled analysis (OR = 1.84, 95% CI = 1.26 to 2.68, *P* = 0.002) from 10 trials. There was increased risk in three olanzapine trials, and no increased risk in one aripiprazole trial, three risperidone trials and three quetiapine trials.

#### Edema

Nine trials reported edema. Increased risks was observed by meta-analysis for edema (OR = 0.63, 95% CI = 0.44 to 0.91, *P* = 0.01). The increased risk was associated with risperidone. Two of three aripiprazole trials, three of five olanzapine trials, four of eight risperidone trials and five of seven quetiapine trials did not report edema.

#### Urinary tract infections

Urinary tract infections were reported in 11 contrasts, including three aripiprazole trials, two olanzapine trials, four risperidone trials and two quetiapine trials. There was overall increased risk for urinary tract infections in the antipsychotic-treated patients (OR = 1.91, 95% CI = 1.48 to 2.46, *P* <0.00001). The effect was not significant with aripiprazole and quetiapine, but was significant when the events were combined. Urinary tract infections were not reported in one olanzapine trial (one trial included risperidone), but urinary incontinence both was and was not reported in the trials of the other drugs.

The article "Efficacy and safety of atypical antipsychotic drug treatment for dementia: a systematic review and meta-analysis" was retracted in 2016. Reasons: errors in the data; errors in the methods.

#### Stroke

Stroke was reported in 13 contrasts including three aripiprazole trials, two olanzapine trials, four risperidone trials and four quetiapine trials. There was overall increased risk for stroke in the antipsychotic-treated patients. Meta-analysis demonstrated a significantly higher risk of stroke in the pooled antipsychotic group (OR = 2.62, 95% CI = 1.45 to 4.75, *P* = 0.001) and in the risperidone subgroup (*P* = 0.002). However, the effect was not significant with aripiprazole, olanzapine and quetiapine (see Additional file 11).

#### Deaths

The overall OR by meta-analysis for death in patients treated with antipsychotics compared with placebo was 1.06 (95% CI = 0.65 to 1.73; *Z* = 0.24, *P* = 0.81). There was no increased risk of death with any individual drug. Besides, in most studies, adverse reactions occurring in less than 20% of patients were not taken into account when not finding a significantly higher prevalence of mortality.

#### All-cause dropouts

In overall meta-analyses on safety, there were no significant differences in the number of dropouts caused by any reason between any medicine treatment group and placebo treatment group (OR = 0.95, 95% CI = 0.82 to 1.09; *Z* = 0.75, *P* = 0.45). In subgroups, we observed similar results (aripiprazole, 95% CI = 0.63 to 1.39; olanzapine, 95% CI = 0.57 to 1.13; risperidone, 95% CI = 0.79 to 1.22; quetiapine, 95% CI = 0.74 to 1.36) (see Additional file 12).

## Discussion

Psychiatric symptoms occur on average in 70% of dementia patients during the primary illness [6]. The use of atypical antipsychotic medications is therefore increasing rapidly. Atypical antipsychotics have been considered preferred pharmacologic treatments for behavioral disturbances associated with dementia because of clinical trial evidence for perceived safety advantages compared with other medications and expert clinical opinion. However, the role of currently available atypical antipsychotics for dementia has been controversial and health economists always question whether the small clinical effects are economically worthwhile. In our present study, we have obtained the treatment effects of 23 trials including 5,819 patients with dementia. Our results show obvious benefits for symptomatic efficacy on psychiatric symptoms and cognitive functions of aripiprazole and risperidone after statistically combining the trials. The safety of atypical antipsychotics may offset the usage of drugs.

A previous study by Schneider and colleagues analyzed 15 RCTs (from published articles or presentations at medical meetings) of three aripiprazole trials, five olanzapine trials, three quetiapine trials and four risperidone and found modest benefits for aripiprazole and risperidone, but also that adverse events and dropouts blocked their efficacy [32]. Furthermore, Maher and colleagues conducted a meta-analysis on efficacy and comparative effectiveness of atypical antipsychotics for off-label uses in psychosis, agitation and global behavioral symptoms in dementia. They found small but statistically significant pooled effect size for aripiprazole, olanzapine and risperidone [33]. A previous paper indicated that aripiprazole shows modest efficacy in the treatment of AD-related psychosis [34]. The benefit of aripiprazole in dementia was consistent in the previous study and our meta-analysis. However, olanzapine was not associated with efficacy overall in our study. Besides, there was a lack of evidence for or against quetiapine because five among the seven trials were dose-ranging and used different selection criteria. The outcomes could not be statistically combined using a common rating scale. Furthermore, Katz and colleagues found that risperidone showed improvement in psychotic symptoms and general clinical improvement in patients with psychosis of AD [28]. However, in our study, risperidone showed improvement in behavior symptoms on dementia. In addition, aripiprazole, olanzapine and quetiapine were more effective for particular symptoms, such as anger and aggression. They all proved to have significant effect on neuropsychiatric symptoms in early studies. As a result, our study is in line with findings from a former review [32] and long-standing clinical experience.

The article "Efficacy and safety of atypical antipsychotic drug treatment for dementia: a systematic review and meta-analysis" was retracted in 2016. Reasons: errors in the data; errors in the methods.

The duration of RCTs of atypical antipsychotics varies from 6 to 26 weeks. Because the length of treatment as well as methodological factors may be stronger outcome modifiers, a considerable number of placebo-controlled RCTs of atypical antipsychotics for stabilizing or slowing decline in psychiatric symptoms and cognitive functions of patients with dementia have been undertaken for generally 6 to 12 weeks in this study. The possible methodological factors that may be relevant as strong outcome modifiers are publication bias or different randomization methods. We only focused on published English-language studies and there are additional unpublished studies that have been identified, which may have introduced a publication bias in favor of studies showing benefits with medications [32]. In addition, although the studies included were randomized, they may not apply the same randomization method.

Safety is as important as the efficacy of the interventions in clinical studies. The five main adverse events were analyzed here and the pooled study showed evidence in increasing somnolence, edema, urinary infection and abnormal gait. Patients receiving atypical antipsychotics showed no difference in risk for injuries or falls (*P* >0.05), and significantly higher risks (*P* <0.05) for somnolence, urinary tract infection or urinary incontinence, edema and abnormal gait. Notably, risperidone had a higher risk on adverse events. However, no drugs improved or aggravated injuries or falls compared with placebos. These events were usually of mild or moderate severity, and the risk disappeared on serious adverse events. Finally, none of these drugs seemed to increase the risk of death in this study, yet the difference did not achieve statistically significant levels. Similarly, Schneider and colleagues found a significant risk for somnolence, abnormal gait, edema, urinary tract infection or urinary incontinence on atypical antipsychotics versus placebo [32]. In general, the results of our meta-analysis demonstrated statistical increased risks of 1.1-fold to 1.5-fold for these adverse events. Thus, an increased risk of AEs in atypical antipsychotics is observed during these years. Importantly, a follow-up study indicated that there was an increased long-term risk of mortality in patients with AD who are prescribed antipsychotic medication [35]. These results further supported the need to seek less harmful alternatives for the long-term treatment of neuropsychiatric symptoms in dementia patients.

The article "Efficacy and safety of atypical antipsychotic drug treatment for dementia: a systematic review and meta-analysis" was retracted in 2016. Reasons: errors in the data; errors in the methods.

Although previous systematic reviews or meta-analysis have been reported, atypical antipsychotics produced modest benefits on neuropsychiatric outcomes. To date, we perform a more comprehensive analysis covering a variety of outcome domains that included many previous studies without a higher risk of bias. Besides, we identified and included five recent studies to conduct an updated meta-analysis, and our results further supported this. There was some evidence to support the efficacy of the atypical antipsychotics when compared with placebo on change in neuropsychiatric symptom scores in the previous reviews [36,37]. These trials offered updated information of atypical antipsychotics in psychiatric symptoms and cognitive functions, which may have contributed to the differences between our review and previous reviews. More importantly, compared with the previous reviews, our study added quality assessment analysis. Quality assessment by GRADE software was used to establish the robustness of the primary outcome, and higher robustness means study drugs have more definite effects on the diseases. Because the magnitude of statistical effect does not always imply a similar magnitude clinical effect, we also reviewed and analyzed each drug separately and by specific outcomes to better address the psychiatric symptoms (see Additional files 13, 14, 15 and 16).

The article "Efficacy and safety of atypical antipsychotic drug treatment for dementia: a systematic review and meta-analysis" was retracted in 2016. Reasons: errors in the data; errors in the methods.

Several limitations to our meta-analysis restrict the interpretation of our results. First, some of our included trials excluded participants receiving psychotropic medicines, while some trials allowed, and even demanded, the use of medicines such as cholinesterase inhibitors and other drugs in their study. The use of such medicines may have an impact on our results. In addition, dementia is progressive and patients declined at progressive different stages of severity, which may also influence our results when pooling data. Finally, there still were very limited trials per each study drug and dose in this present study; unfortunately, some items tested in the trials were not available in the results, and despite numerous attempts to contact the authors, further details were still absent. In addition, we must note that despite differences in outcome measures such as the NPI and so forth, the outcome symptoms may also differ among studies (such as agitation and/of psychosis). Therefore, no convincing conclusions can be drawn regarding the efficacy of these drugs for neuropsychiatric symptoms. Furthermore, some trials found no significant differences in outcomes between the withdrawal of the drugs and continuation groups. Decision-making related to antipsychotic drug treatment in dementia remains challenging and requires a thoughtful approach [38]. What is worth noting is that the heterogeneity was substantial for the outcomes. We detected a substantial heterogeneity in meta-analyses in NPI psychosis or BPRS psychosis. There are several interpretations for the heterogeneity. First, it may indicate that many differences still exist between different kinds of dementia, although they are highly identical in clinical and neuropathological symptoms. The second sources of heterogeneity may be the discrepancy in treatment duration and bias risk, and the diversity in concomitant pathologic condition and drug therapy.

Despite some limitations, we believe that our results are the newest and most comprehensive attempt to quantitatively synthesize the efficacy and safety of atypical antipsychotics for neuropsychiatric symptoms of dementia patients, suggesting a moderate benefit in neuropsychiatric outcomes from antipsychotics. Our meta-analysis results indicate that for dementia patients who have neuropsychiatric disturbances, atypical antipsychotics may be considered as a therapeutic option. However, it is notable that the decision to use these medicines needs to be considered in light of the adverse effects, cost and feasibility. As recommended, for dementia patients with neuropsychiatric symptoms, excluding medical and environmental factors, drug therapy should be used to manage neuropsychiatric symptoms. Overall, our meta-analysis results indicate a benefit in neuropsychiatric symptoms for dementia patients from atypical antipsychotics.

The article "Efficacy and safety of atypical antipsychotic drug treatment for dementia: a systematic review and meta-analysis" was retracted in 2016. Reasons: errors in the data; errors in the methods.

## Conclusion

Obvious benefits were observed for symptomatic efficacy on psychiatric symptoms and cognitive functions of aripiprazole and risperidone after statistically combining the trials. The higher risks for adverse events may offset the efficacy of atypical antipsychotics for treatment of dementia. Hopefully, the design of a multicenter study could use currently available levels of treatment and care, in order to provide a broader generalizability of the results in the future. Future research should focus more on neuropsychiatric outcomes. It is important to continue efforts to perform high-quality trials of drug therapy, and the safety evaluation of the drugs cannot be ignored.

## Additional files

Additional file 1:
**Is a table presenting the basic information of all included studies.**
Additional file 2:
**Is a forest plot of specific BPRS psychosis subscales on dementia patients in subgroup analyses.** Data type, continuous; effect measure, weighted mean difference; analysis model, fixed effects; statistical method, inverse variance. Additional file 3:
**Is a forest plot of specific NPI psychosis subscales on dementia patients in subgroup analyses.** Data type, continuous; effect measure, weighted mean difference; analysis model, fixed effects; statistical method, inverse variance. Additional file 4:
**Is a forest plot of specific BEHAVE-AD psychosis subscales on dementia patients in subgroup analyses.** Data type, continuous; effect measure, weighted mean difference; analysis model, fixed effects; statistical method, inverse variance. Additional file 5:
**Is a table presenting the quality assessment on NPI of all included studies in dementia patients.**
Additional file 6:
**Is a table presenting the quality assessment on BPRS of all included studies in dementia patients.**
Additional file 7:
**Is a table presenting the quality assessment on BEHAVE-AD of all included studies in dementia patients.**
Additional file 8:
**Is a table presenting the quality assessment on CGI-C of all included studies in dementia patients.**
Additional file 9:
**Is a table presenting the quality assessment on MMSE of all included studies in dementia patients.**
Additional file 10:
**Is a table presenting the quality assessment on adverse events of all included studies in dementia patients.**
Additional file 11:
**Is a forest plot of stroke of four drugs on all-cause dropouts in dementia patients.** Data type, dichotomous; effect measure, odds ratio; analysis model, fixed effects; statistical method, Mantel–Haenszel. Additional file 12:
**Is a forest plot of safety of four drugs on all-cause dropouts in dementia patients.** Data type, dichotomous; effect measure, odds ratio; analysis model, fixed effects; statistical method, Mantel–Haenszel. Additional file 13:
**Is a forest plot of aripiprazole on dementia patients in subgroup analyses.** Data type, continuous; effect measure, weighted mean difference; analysis model, fixed effects; statistical method, inverse variance. Additional file 14:
**Is a forest plot of olanzapine on dementia patients in subgroup analyses.** Data type, continuous; effect measure, weighted mean difference; analysis model, fixed effects; statistical method, inverse variance. Additional file 15:
**Is a forest plot of quetiapine on dementia patients in subgroup analyses.** Data type, continuous; effect measure, weighted mean difference; analysis model, fixed effects; statistical method, inverse variance. Additional file 16:
**Is a forest plot of risperidone on dementia patients in subgroup analyses.** Data type, continuous; effect measure, weighted mean difference; analysis model, fixed effects; statistical method, inverse variance.

The article "Efficacy and safety of atypical antipsychotic drug treatment for dementia: a systematic review and meta-analysis" was retracted in 2016. Reasons: errors in the data; errors in the methods.

## Abbreviations

AD: Alzheimer’s disease
BEHAVE-AD: Behavioral Pathology in Alzheimer’s Disease Rating Scale
BPRS: Brief Psychiatric Rating Scale
CGI-C: Clinical Global Impression –Change
CGI-S: Clinical Global Impression – Severity
CI: confidence interval
CMAI: Cohen-Mansfield Agitation Inventory
MMSE: Minimum Mental State Examination
NPI: Neuropsychiatric Inventory
OR: odds ratio
RCT: randomized controlled trial
WMD: weighted mean difference

## References

[1] Jeste DV, Finkel SI (2000). Psychosis of Alzheimer's disease and related dementias. Diagnostic criteria for a distinct syndrome. Am J Geriatr Psychiatry.

[2] Butler R, Radhakrishnan R. Dementia. Clin Evid (Online). 2012;2012:1001.PMC343752623870856

[3] Declercq T, Petrovic M, Azermai M, Vander Stichele R, De Sutter AI, van Driel ML (2013). Withdrawal versus continuation of chronic antipsychotic drugs for behavioural and psychological symptoms in older people with dementia. Cochrane Database Syst Rev..

[4] Alexopoulos GS, Jeste DV, Chung H, Carpenter D, Ross R, Docherty JP. The expert consensus guideline series. Treatment of dementia and its behavioral disturbances. Introduction: methods, commentary, and summary. Postgrad Med. 2005;Spec No:6–22.17203561

[5] Sink KM, Holden KF, Yaffe K (2005). Pharmacological treatment of neuropsychiatric symptoms of dementia: a review of the evidence. JAMA..

The article "Efficacy and safety of atypical antipsychotic drug treatment for dementia: a systematic review and meta-analysis" was retracted in 2016. Reasons: errors in the data; errors in the methods.

[6] Ballard C, Waite J (2006). The effectiveness of atypical antipsychotics for the treatment of aggression and psychosis in Alzheimer's disease. Cochrane Database Syst Rev.

[7] Cooper JE (1995). On the publication of the Diagnostic and Statistical Manual of Mental Disorders: Fourth Edition (DSM-IV). Br J Psychiatry.

[8] Overall JE, Beller SA (1984). The Brief Psychiatric Rating Scale (BPRS) in geropsychiatric research: I. Factor structure on an inpatient unit. J Gerontol.

[9] Cummings JL, Mega M, Gray K, Rosenberg-Thompson S, Carusi DA, Gornbein J (1994). The Neuropsychiatric Inventory: comprehensive assessment of psychopathology in dementia. Neurology..

[10] Reisberg B, Borenstein J, Salob SP, Ferris SH, Franssen E, Georgotas A (1987). Behavioral symptoms in Alzheimer's disease: phenomenology and treatment. J Clin Psychiatry..

[11] Cohen-Mansfield J, Marx MS, Rosenthal AS (1989). A description of agitation in a nursing home. J Gerontol..

[12] Schneider LS, Olin JT, Doody RS, Clark CM, Morris JC, Reisberg B (1997). Validity and reliability of the Alzheimer's Disease Cooperative Study–Clinical Global Impression of Change. The Alzheimer's Disease Cooperative Study. Alzheimer Dis Assoc Disord..

[13] Higgins JPT, Green S (editors). Cochrane Handbook for Systematic Reviews of Interventions Version 5.1.0 [updated March 2011]. The Cochrane Collaboration. 2011. www.cochrane-handbook.org.

[14] Streim JE, Porsteinsson AP, Breder CD, Swanink R, Marcus R, McQuade R (2008). A randomized, double-blind, placebo-controlled study of aripiprazole for the treatment of psychosis in nursing home patients with Alzheimer disease. Am J Geriatr Psychiatry..

[15] Mintzer JE, Tune LE, Breder CD, Swanink R, Marcus RN, McQuade RD (2007). Aripiprazole for the treatment of psychoses in institutionalized patients with Alzheimer dementia: a multicenter, randomized, double-blind, placebo-controlled assessment of three fixed doses. Am J Geriatr Psychiatry..

[16] De Deyn P, Jeste DV, Swanink R, Kostic D, Breder C, Carson WH (2005). Aripiprazole for the treatment of psychosis in patients with Alzheimer's disease: a randomized, placebo-controlled study. J Clin Psychopharmacol..

[17] Sultzer DL, Davis SM, Tariot PN, Dagerman KS, Lebowitz BD, Lyketsos CG (2008). Clinical symptom responses to atypical antipsychotic medications in Alzheimer's disease: phase 1 outcomes from the CATIE-AD effectiveness trial. Am J Psychiatry..

[18] Street JS, Clark WS, Gannon KS, Cummings JL, Bymaster FP, Tamura RN (2000). Olanzapine treatment of psychotic and behavioral symptoms in patients with Alzheimer disease in nursing care facilities: a double-blind, randomized, placebo-controlled trial. The HGEU Study Group. Arch Gen Psychiatry..

The article "Efficacy and safety of atypical antipsychotic drug treatment for dementia: a systematic review and meta-analysis" was retracted in 2016. Reasons: errors in the data; errors in the methods.

[19] Schneider LS, Tariot PN, Dagerman KS, Davis SM, Hsiao JK, Ismail MS (2006). Effectiveness of atypical antipsychotic drugs in patients with Alzheimer's disease. N Engl J Med..

[20] Deberdt WG, Dysken MW, Rappaport SA, Feldman PD, Young CA, Hay DP (2005). Comparison of olanzapine and risperidone in the treatment of psychosis and associated behavioral disturbances in patients with dementia. Am J Geriatr Psychiatry..

[21] De Deyn PP, Carrasco MM, Deberdt W, Jeandel C, Hay DP, Feldman PD (2004). Olanzapine versus placebo in the treatment of psychosis with or without associated behavioral disturbances in patients with Alzheimer's disease. Int J Geriatr Psychiatry..

[22] Zhong KX, Tariot PN, Mintzer J, Minkwitz MC, Devine NA (2007). Quetiapine to treat agitation in dementia: a randomized, double-blind, placebo-controlled study. Curr Alzheimer Res..

[23] Tariot PN, Schneider L, Katz IR, Mintzer JE, Street J, Copenhaver M (2006). Quetiapine treatment of psychosis associated with dementia: a double-blind, randomized, placebo-controlled clinical trial. Am J Geriatr Psychiatry..

[24] Paleacu D, Barak Y, Mirecky I, Mazeh D (2008). Quetiapine treatment for behavioural and psychological symptoms of dementia in Alzheimer's disease patients: a 6-week, double-blind, placebo-controlled study. Int J Geriatr Psychiatry..

[25] Kurlan R, Cummings J, Raman R, Thal L (2007). Quetiapine for agitation or psychosis in patients with dementia and parkinsonism. Neurology..

[26] Ballard C, Margallo-Lana M, Juszczak E, Douglas S, Swann A, Thomas A (2005). Quetiapine and rivastigmine and cognitive decline in Alzheimer's disease: randomised double blind placebo controlled trial. BMJ..

[27] Mintzer J, Greenspan A, Caers I, Van Hove I, Kushner S, Weiner M (2006). Risperidone in the treatment of psychosis of Alzheimer disease: results from a prospective clinical trial. Am J Geriatr Psychiatry..

[28] Katz IR, Jeste DV, Mintzer JE, Clyde C, Napolitano J, Brecher M (1999). Comparison of risperidone and placebo for psychosis and behavioral disturbances associated with dementia: a randomized, double-blind trial. Risperidone Study Group. J Clin Psychiatry..

[29] De Deyn PP, Rabheru K, Rasmussen A, Bocksberger JP, Dautzenberg PL, Eriksson S (1999). A randomized trial of risperidone, placebo, and haloperidol for behavioral symptoms of dementia. Neurology..

[30] Brodaty H, Ames D, Snowdon J, Woodward M, Kirwan J, Clarnette R (2003). A randomized placebo-controlled trial of risperidone for the treatment of aggression, agitation, and psychosis of dementia. J Clin Psychiatry..

[31] Brodaty H, Ames D, Snowdon J, Woodward M, Kirwan J, Clarnette R (2005). Risperidone for psychosis of Alzheimer's disease and mixed dementia: results of a double-blind, placebo-controlled trial. Int J Geriatr Psychiatry..

The article "Efficacy and safety of atypical antipsychotic drug treatment for dementia: a systematic review and meta-analysis" was retracted in 2016. Reasons: errors in the data; errors in the methods.

[32] Schneider LS, Dagerman K, Insel PS (2006). Efficacy and adverse effects of atypical antipsychotics for dementia: meta-analysis of randomized, placebo-controlled trials. Am J Geriatr Psychiatry..

[33] Maher AR, Maglione M, Bagley S, Suttorp M, Hu JH, Ewing B (2011). Efficacy and comparative effectiveness of atypical antipsychotic medications for off-label uses in adults: a systematic review and meta-analysis. JAMA..

[34] De Deyn PP, Drenth AF, Kremer BP, Oude Voshaar RC, Van Dam D (2013). Aripiprazole in the treatment of Alzheimer's disease. Expert Opin Pharmacother..

[35] Ballard C, Hanney ML, Theodoulou M, Douglas S, McShane R, Kossakowski K (2009). The dementia antipsychotic withdrawal trial (DART-AD): long-term follow-up of a randomised placebo-controlled trial. Lancet Neurol..

[36] Seitz DP, Gill SS, Herrmann N, Brisbin S, Rapoport MJ, Rines J (2013). Pharmacological treatments for neuropsychiatric symptoms of dementia in long-term care: a systematic review. Int Psychogeriatr..

[37] Franco KN, Messinger-Rapport B (2006). Pharmacological treatment of neuropsychiatric symptoms of dementia: a review of the evidence. J Am Med Dir Assoc..

[38] Gill SS, Seitz DP (2013). Antipsychotics can be withdrawn from many older people with dementia, though caution is needed for people with more severe neuropsychiatric symptoms. Evid Based Ment Health..

